# Risk Factors and Risk Model Construction of Stroke in Patients with Vertigo in Emergency Department

**DOI:** 10.1155/2022/2968044

**Published:** 2022-05-20

**Authors:** Zhuqing Zhu, Qian Li, Li Wang, Chunling Xiao, Hui Wang, Yan Xu

**Affiliations:** ^1^Jiangsu Food & Pharmaceutical Science College, Huai'an, Jiangsu 223023, China; ^2^Department of Emergency, Huai'an Second People's Hospital, Huai'an, Jiangsu 223001, China; ^3^Department of Nursing, Huai'an Second People's Hospital, Huai'an, Jiangsu 223001, China

## Abstract

**Objective:**

We aimed to explore the risk factors of stroke in patients with vertigo in the emergency department and establish a risk prediction model for stroke patients.

**Methods:**

A total of 301 patients experiencing vertigo in our hospital from January 2020 to January 2021 were retrospectively included. Patients were divided into the stroke group (*n* = 56) and the nonstroke group (*n* = 245). The clinical characteristics of patients in both groups were collected and compared, followed by binary logistic regression that was employed to determine the risk factors that affect stroke diagnosis. The receiver operating characteristic (ROC) curve was used to clarify the effectiveness of the constructed model.

**Results:**

Patients in the stroke group were older and had higher systolic and diastolic blood pressure on admission than the nonstroke group. Meanwhile, they demonstrated a higher proportion of diabetes and atrial fibrillation and focal muscle weakness, dysarthria, dysphagia, or ataxia in neurological examinations compared to the nonstroke group (all *P* < 0.05). The proportion of patients in the nonstroke group who had a history of vertigo or inner ear disease was significantly higher than that in the stroke group (*P* < 0.05). The patient's age ≥ 60 years old (OR = 3.57), diabetes (OR = 4.57), atrial fibrillation (OR = 4.26), previous history of vertigo or inner ear disease (OR = 0.16), focal muscle weakness (OR = 4.34), and dysphagia or ataxia (OR = 4.08) were associated with a higher risk of stroke. The area under the curve for stroke was 0.87, and the sensitivity and specificity were 98.2% and 57.6%, respectively, as the sum of the assigned scores was greater than 3.

**Conclusions:**

Age ≥ 60 years old, diabetes, atrial fibrillation, previous history of vertigo or inner ear disease, focal muscle weakness, dysphagia, or ataxia were associated with a higher risk of stroke. The risk model constructed based on our findings may help to assess the risk of stroke in patients with vertigo in the emergency department.

## 1. Introduction

Vertigo is common complaints seen in the emergency department. Studies have found that the primary cause of up to 4% of emergency department visits is vertigo [1]. The causes of vertigo are diverse, including otolith, Meniere's syndrome, vertebrobasilar insufficiency, and moderate stroke, thus making the diagnosis of vertigo very difficult [2]. Meanwhile, vertigo caused by stroke often progresses rapidly. Early detection and intervention can significantly improve the prognosis of patients. Therefore, distinguishing between stroke and nonstroke in the emergency room is of great clinical significance. At present, the ABCD2 score is widely used to determine whether vertigo patients have stroke preliminarily. The standard for evaluation mainly includes five aspects: age, blood pressure, clinical presentation, duration of symptoms, and diabetes [3]. However, the score comes from the population with a transient ischemic attack, and the prediction efficiency of stroke caused by macrovascular disease is poor [4]. This study retrospectively analyzed the clinical data of vertigo patients in the emergency department of our hospital, identified the risk factors related to the diagnosis of stroke, and constructed a risk model.

## 2. Materials and Methods

### 2.1. Research Object

This study retrospectively included 301 patients in the emergency department of our hospital with “vertigo” as the first symptom from January 2020 to January 2021. Inclusion criteria: (1) the first medical record was “vertigo”; (2) the cause was finally diagnosed. Exclusion criteria: (1) the patient had an apparent history of trauma and bleeding before seeing a doctor; (2) incomplete records of medical history and vital signs and lack of admission blood pressure and other records; (3) patients with final vertigo without definite diagnosis; (4) the patient had no cranial imaging results and could not determine whether there was a stroke.

### 2.2. Research Methods

The clinical and imaging data of patients presenting to the emergency department were collected through the electronic medical record system, including patient age, gender, systolic blood pressure, diastolic blood pressure complications (hypertension, diabetes, hyperlipidemia, coronary atherosclerotic heart disease, and atrial fibrillation), smoking, past stroke/transient ischemic attack, past vertigo and inner ear history, current use of antiplatelet and anticoagulant drugs, combined symptoms (headache, shoulder pain, ear distention, or hearing loss), and neurological findings (focal hyperdynamic, dysarthria, nystagmus, dysphagia, and ataxia) according to the final diagnosis. The patients were divided into stroke group and nonstroke group.

### 2.3. Statistical Analysis

SPSS 24.0 Chinese version software was used for statistical analysis. The measurement data of nonnormal distribution were expressed by the median and interquartile range (IQR). The groups were compared using the Mann–Whitney *U* nonparametric test. The counting data were expressed in frequency and percentage, and the groups were compared by the chi-square test. Bring the statistically significant variables in the univariate comparison into the binary logistic regression analysis and take whether the patient has a stroke as the dependent variable to clarify the variables affecting the patient's stroke. Each meaningful variable was assigned according to the obtained risk ratio. The assigned variables were identified by the subject's working characteristic curve to determine whether the patient was the best cut value, the area under the curve (AUC), sensitivity, and specificity of stroke. Bilateral test, test level *α* = 0.05.

## 3. Results

### 3.1. Comparison of General Characteristics of Patients

Of the 301 patients included in this study, 56 were diagnosed with a stroke, and 245 were nonstroke. Compared with the nonstroke group, the stroke group had higher age, a higher systolic and diastolic blood pressure, a higher proportion of diabetes and atrial fibrillation, and focal muscle weakness and dysarthria in the neurological examination. The positive rate of dysphagia or ataxia was higher (all *P* < 0.05). The proportion of patients with a previous history of vertigo or inner ear in the nonstroke group was significantly higher than that in the stroke group (*P* < 0.05), see Table 1.

### 3.2. Multivariate Logistic Regression Analysis

All statistically significant variables in Table 1 were brought into binary logistic regression for analysis. It was found that patients aged over 60 years (OR = 3.57), diabetes mellitus (OR = 4.57), atrial fibrillation (OR = 4.26), past vertigo or inner ear history (OR = 0.16), focal muscular weakness (OR = 4.34), and dysphagia or ataxia (OR = 4.08) were associated with a higher risk of stroke, as shown in Table 2.

### 3.3. Assignment of Relevant Factors

According to the results in Table 2, the corresponding statistically significant indicators were assigned, and the results were shown in Table 3. The previous history of vertigo or inner ear was the protective factor of stroke, with a value of -6 (1/0.16), and the other factors were harmful factors, with a positive value.

### 3.4. ROC Curve

The results of the ROC curve showed that when the total score of patients was >3, the AUC of stroke in vertigo patients was 0.87 (95% CI, 0.82-0.90), and the sensitivity and specificity were 98.2% and 57.6%, respectively, as shown in Figure 1. When the total score of patients was >13, the specificity of stroke in vertigo patients was as high as 100%.

## 4. Discussion

Vertigo is one of the main complaints often encountered by medical staff in the emergency department in clinical work. There are various causes of vertigo, and some patients have benign outcomes. In this study, we identified stroke risk factors in 301 patients with “vertigo” and constructed the related risk model.

This study found that age ≥ 60 was associated with the risk of being diagnosed with “stroke” in patients with vertigo, which was consistent with previous reports. A previous [5] stroke-related epidemiologic study suggested that the incidence rate of stroke in adults aged 35-44 years was 30-120/100000 per year, while the incidence rate in 65-74 years olds increased significantly to 670-970/100000 per year. Kerber and his colleagues' study of 1666 patients with vertigo in the emergency department showed that the average age of patients finally diagnosed with stroke was significantly higher than patients without stroke [6]. It suggests that medical staff should pay special attention to excluding the possibility of stroke when receiving elderly patients with vertigo.

Similar to previous studies, this study also found that diabetes in stroke patients was significantly higher than that in nondiabetic patients. Diabetes and other metabolic abnormalities have been recognized as risk factors for stroke [7, 8]. Lee et al. found that diabetes mellitus can significantly increase the risk of stroke in hospitalized vertigo patients [9].

This study found that atrial fibrillation was associated with a higher risk of stroke in patients with vertigo diagnosed with stroke. Long-term atrial fibrillation will produce mural thrombus, which will enter the brain with blood flow after falling off, resulting in ischemic stroke [10, 11]. After analyzing the data of Denmark, Christiansen et al. [12] found that the incidence of stroke with atrial fibrillation in the 50-year-old population was 1.1%. If the patient had a history of stroke before, the risk of stroke recurrence within 5 years was 10.2%.

The previous history of vertigo or inner ear is a protective factor in diagnosing stroke in patients with vertigo. In other words, if the patient has recurrent vertigo or has a clear history of the inner ear, the possibility of vertigo caused by stroke will be reduced. A single-center retrospective study conducted by Kuroda et al. [13] found that no previous history of vertigo or inner ear can significantly increase the risk of stroke in vertigo patients. It suggests that it is crucial for medical staff in the emergency department to inquire about the history of vertigo or inner ear in detail.

Positive neurological signs, including focal hypodynamia, dysphagia, and ataxia, are crucial for diagnosing stroke. In the classic ABCD2 scoring system, the clinical manifestation (c) is unilateral weakness and language disorder, with 2 and 1 points, respectively [4]. Navi et al. found that the ABCD2 scoring system is helpful to assist in identifying vertigo patients in the emergency department as stroke [14].

This study has some limitations. First, this study is a retrospective analysis, so the possible bias will affect the results and conclusions of the study. Second, this study is designed as a single-center, and the models and findings need to be confirmed by prospective and multicenter studies. Finally, due to the differences in the characteristics of the population included in different research institutes, this study may not apply to other characteristic populations.

To sum up, this study explored stroke risk factors in patients with vertigo in the emergency department and established a risk prediction model. It was found that age over 60 years old, diabetes mellitus, atrial fibrillation, history of vertigo or inner ear disease, focal muscle strength reduction, dysphagia, or ataxia were associated with a higher risk of stroke. The model constructed in this study may be helpful for medical staff in the emergency department to identify patients with vertigo caused by stroke in clinical work.

## Figures and Tables

**Figure 1:** Working characteristic curve of subjects with the total score assigned to identify whether vertigo patients are stroke.

**Table 1:** Comparison of general characteristics between stroke group and nonstroke group.

	Stroke group (*n* = 56)	Nonstroke group (*n* = 245)	*χ* ^2^/*Z* value	*P* value
Age (years) (IQR)	70 (59, 78)	54 (44, 66)	-5.44	<0.001
Age ≥ 60 years (cases, %)	39 (69.64)	93 (37.96)	18.58	<0.001
Gender (male) (cases, %)	27 (48.21)	91 (37.14)	2.34	0.13
Systolic blood pressure (mmHg) (IQR)	157 (140.25, 175)	137 (124, 154.50)	-5.45	<0.001
Diastolic blood pressure (mmHg) (IQR)	90.5 (76.5, 98.0)	79 (71, 89.5)	-3.69	<0.001
Systolic blood pressure ≥ 140/diastolic blood pressure ≥ 90 mmHg (cases, %)	44 (78.57)	115 (46.94)	18.30	<0.001
Complication				
Hypertension (cases, %)	37 (66.07)	132 (53.88)	2.75	0.10
Diabetes mellitus (case, %)	35 (57.14)	67 (27.35)	25.14	<0.001
Hyperlipidemia (cases, %)	25 (44.64)	106 (43.27)	0.04	0.85
Coronary atherosclerotic heart disease (cases, %)	8 (14.29)	36 (14.69)	2.63	0.11
Atrial fibrillation (cases, %)	12 (21.43)	13 (5.31)	15.56	<0.001
Smoking (cases, %)	26 (46.43)	105 (42.86)	0.24	0.63
Previous history of stroke/transient ischemic attack (cases, %)	7 (12.50)	17 (6.94)	1.92	0.17
Previous history of vertigo or inner ear (cases, %)	5 (8.93)	92 (37.55)	17.10	<0.001
Currently used drugs				
Antiplatelet drugs (cases, %)	13 (23.21)	62 (25.31)	0.11	0.74
Anticoagulant drugs (cases, %)	4 (7.14)	21 (8.57)	0.12	0.73
Combined symptoms				
Headache or shoulder pain (cases, %)	5 (8.93)	23 (9.39)	0.01	0.92
Ear distention or hearing loss (cases, %)	7 (12.50)	29 (11.84)	0.02	0.89
Nervous system examination				
Focal hypodynamia (cases, %)	25 (44.64)	34 (13.88)	27.38	<0.001
Dysarthria (cases, %)	14 (25.00)	24 (9.80)	9.55	0.002
Nystagmus (cases, %)	6 (10.71)	23 (9.39)	0.09	0.76
Dysphagia or ataxia (cases, %)	17 (30.36)	28 (11.43)	12.84	<0.001

IQR: interquartile range.

**Table 2:** Results of multivariate binary logistic regression analysis for predicting stroke in patients with vertigo.

Factors	*β*	SE	Wald	*P* value	OR value (95% CI)
Age (≥60 years = 1; <60 years = 0)	1.27	0.41	9.61	0.002	3.57 (1.60, 7.97)
Systolic blood pressure (≥140 mmHg = 1; <140 mmHg = 0)	0.88	0.49	3.25	0.07	2.41 (0.93, 6.27)
Diastolic blood pressure (≥90 mmHg = 1; <90 mmHg = 0)	0.34	0.45	0.58	0.45	1.41 (0.58, 3.41)
Diabetes mellitus (with = 1; no = 0)	1.52	0.40	14.75	<0.001	4.57 (2.10, 9.91)
Atrial fibrillation (yes = 1; no = 0)	1.45	0.57	6.59	0.01	4.26 (1.41, 12.89)
Previous history of vertigo or inner ear (yes = 1; no = 0)	-1.83	0.57	10.36	0.001	0.16 (0.05, 0.49)
Focal hypodynamia (yes = 1; no = 0)	1.47	0.41	12.72	<0.001	4.34 (1.94, 9.74)
Dysarthria (yes = 1; no = 0)	0.95	0.50	3.54	0.06	2.58 (0.96, 6.91)
Dysphagia or ataxia (yes = 1; no = 0)	1.41	0.47	8.94	0.003	4.08 (1.62, 10.25)

CI: confidence interval; OR: odds ratio; SE: standard error.

**Table 3:** Evaluation of risk factors for stroke in patients with vertigo.

Variable	Assignment
Age ≥ 60 years	4
Diabetes mellitus	5
Atrial fibrillation	4
Previous history of vertigo or inner ear	-6
Focal hypodynamia	4
Dysphagia or ataxia	4

## Data Availability

The data used to support the findings of this study are included within the article.
